This article has been retracted.

# Changes in T-Cell Subsets and Serum IFN-*γ*, IL-17, and IgE Levels in Children with Respiratory Syncytial Virus Capillary Bronchitis and Their Clinical Significance

**DOI:** 10.1155/2022/2549845

**Published:** 2022-10-12

**Authors:** Yao Zhang, Jianfeng Luo, Huajie Wu, Hao Wang, Xin Sun

**Affiliations:** Pediatrics Department, Xijing Hospital Affiliated to Xi'an Air Force Military Medical University, China

## Abstract

**Objective:**

To investigate the changes in T-cell subsets and serum IFN-*γ*, IL-17, and IgE levels in children with respiratory syncytial virus capillary bronchitis and their clinical significance.

**Methods:**

The clinical data of 50 children with respiratory syncytial virus capillary bronchitis admitted to our hospital between July 2020 and June 2021 were retrospectively reviewed, and they were included in the observation group, while 50 children with a healthy physical examination during the same period were chosen as the control group. The T-cell subsets (CD4, CD8, and CD4/CD8) and serum IL-4, IL-8, IFN-, IL-17, and IgE levels of children in the two groups were compared, and the clinical significance of the changes in the levels of the indices mentioned above was analyzed.

**Results:**

There was no statistically significant difference in T-cell subset levels (CD4 and CD8) between the two groups (*P* > 0.05); the level of CD4/CD8, IL-4, IL-8, IL-17, and IgE in the observation group were substantially higher than those in the control group (*P* < 0.05), while the serum IFN-*γ* levels in the observation group were significantly lower than those in the control group (*P* < 0.05).

**Conclusion:**

Increased CD4/CD8 levels in children with respiratory syncytial virus capillary bronchitis cause an imbalance in the Th1/Th2 immune response, similar to changes in bronchial asthma, suggesting a link between the two diseases. Increased serum levels of IL-4, IL-8, IL-17, and IgE and decreased serum levels of IFN-*γ* have been seen in children with respiratory syncytial virus capillary bronchitis, suggesting the severity of the children's disease may in part be reflected in the levels of the aforementioned serum indicators.

## 1. Introduction

Bronchiolitis, also known as wheezing pneumonia, is a common clinical respiratory tract infection, mostly in infants under 2 years old. According to epidemiological data, bronchiolitis is an important factor causing bronchial asthma in infants and young children, and it is prone to recurrent wheezing symptoms after treatment, especially for children with atopic constitution. Respiratory syncytial virus (RSV) is one of the most prevalent pathogens causing respiratory infections in clinical pediatrics. Its common infected population is infants and young children, with epidemic outbreaks regularly occurring [1]. Rhinitis and pharyngitis may appear many days after infection, and when the illness develops, children may develop acute capillary bronchitis [2]. Cough, shortness of breath, and dyspnea are symptoms of respiratory syncytial virus capillary bronchitis in children [3], with severe cases displaying acute cardiac insufficiency and acute respiratory failure [4]. According to Wang Qi et al., multiple cytokines are implicated in the pathogenesis of capillary bronchitis in children, and the disease has similar pathogenesis to asthma [5].

As previously reported, IgE and IL-17 are involved in the pathogenesis of bronchiolitis. IgE is a major inflammatory mediator of allergic diseases in the body. Additionally, the level of IgE in the body can reflect the allergic reaction of the body to a large extent. Therefore, the serum IgE level of the patient is often used in clinic to determine the allergic reaction of the patient and make an early diagnosis. IL-17 is also a very important inflammatory mediator, which originates from Th17 cells and is secreted by Th17 cells. According to clinical studies, the level of IL-17 can largely reflect the disease severity of children with bronchiolitis [6]. Scholars Li Mengwan [7] and colleagues discovered that during the pathogenesis of children with capillary bronchitis, their serum IL-4 and IL-8 levels increase dramatically, while their serum IFN-*γ* levels decrease, and there is an abnormal ratio of peripheral blood T lymphocytes in these children, indicating that IL-4, IL-8, IFN-*γ*, and peripheral blood T lymphocytes play a crucial role in the pathogenesis and advancement of children with capillary bronchitis [8]. While immunoglobulin E (IgE) is an immunoglobulin, it is mostly involved in type I allergic reactions, and relevant research has shown that it plays an important role in the occurrence and progression of allergic diseases [9]. INF-*γ* is mainly produced by Th1 cells, and Th0 can also secrete INF-*γ*. Moreover, INF-*γ* is also an important active substance that regulates the balance of Th1/Th2 immune response. Previous studies have found that the level of INF-*γ* in patients with bronchiolitis and asthma can be significantly reduced, leading to Th1/Thl2 imbalance, which in turn leads to increased inflammatory response and activation of eosinophils.

In this study, we retrospectively analyzed the clinical data of 50 children with respiratory syncytial virus capillary bronchitis admitted to our hospital between July 2020 and June 2021, intending to investigate the changes in T-cell subsets and serum IFN-*γ*, IL-17, and IgE levels in children with respiratory syncytial virus capillary bronchitis and their clinical significance in order to give appropriate clinical recommendations.

## 2. Materials and Methods

### 2.1. General Information

The clinical data of 50 children with respiratory syncytial virus capillary bronchitis admitted to our hospital from July 2020 to June 2021 were analyzed retrospectively and included in the observation group, while 50 children with healthy physical examinations during the same period were chosen as the control group. Randomization was undertaken online using a web-based randomization service, achieving full allocation concealment (https://www.sealedenvelope.co.uk). Stratified randomization with random block sizes was used to randomize in a 1 : 1 ratio at the level of the patient, with the stratification factors of diagnosis and treatment center. The observation group included 27 boys and 23 girls ranging in age from 3 to 34 months, with a mean age of 14.52 ± 5.27 months. The control group included 25 boys and 25 girls ranging in age from 4 to 35 months, with a mean age of 14.62 ± 5.18 months.

#### 2.1.1. Sample Size Estimation

The original sample size calculation estimated that 40-50 patients in each group would be needed to detect a 3-point difference between groups in a 2-sided significance test with a power of 0.8 and an alpha error level of 0.05.

#### 2.1.2. Ethical Considerations

The study protocol and all amendments were approved by the appropriate ethics committee at each center. The study was done in accordance with the protocol, its amendments, and standards of Clinical Practice. All participants provided written informed consent before enrolment. Ethics No.:(2020214).

### 2.2. Inclusion and Exclusion Criteria

Participants were assessed eligible if (1) at the time of enrollment, the duration of the disease was less than three days; (2) the diagnostic criteria for clinical respiratory syncytial virus capillary bronchitis were met; (3) the children had not recently been treated; (4) first onset; (5) acute exacerbation of respiratory wheezing; and (6) signs of viral respiratory tract infection;

Participants were assessed ineligible if they had (1) other serious organ diseases that were not eligible; (2) family members who were uncooperative or had poor compliance were not included in the study; (3) Kawasaki disease, inflammatory bowel disease, immune-related diseases, and chronic infectious diseases such as tuberculosis; (4) congenital respiratory malformations or dysplasia; (5) renal insufficiency; and (6) severe pneumonia and malnutrition.

### 2.3. Detection Method

(1) Flow cytometry assay was used to determine the levels of T-cell subsets (CD4, CD8, and CD4/CD8) in the children. The utilized reagents were from a CD4-FITC/CD8-PE/CD3CY5 fluorescently labeled monoclonal antibody kit (trichrome) produced by Immunotech in France. The type of the detection device was Beckman Coulter Epics XL Flow Cytometer. (2) The serum IL-4, IL-8, IL-17, and IFN-*γ* levels of the children were measured by enzyme-linked immunosorbent assay (ELISA). The enzyme immunoassay kit for detecting serum IL-4 and IL-8 levels in children was supplied by Jingmei Biotech Co.; the enzyme immunoassay kit for detecting serum IL-17 levels in children was supplied by R&D in the USA; the enzyme immunoassay kit for detecting serum IFN-*γ* levels in children was supplied by MingRui Biotech Co., Ltd. (3) The serum IgE levels of the children were measured using the chemiluminescence method. The kit for IgE assay was provided by Beckman Coulter Inc. in the USA.

### 2.4. Statistical Methods

The mean difference between the two groups was tested using the Student's *t*-test for normally distributed variables and the Mann–Whitney *U* test for nonnormal variables. SPSS 21.0 was selected as the software for data analysis, and the measurement data were expressed as ±s with an independent sample *t*-test; the count data were expressed as case number (rate) with an *X*^2^ test. *P* < 0.05 indicated that the comparison was statistically significant.

## 3. Results

### 3.1. General Information in the Two Groups

There was no statistically significant difference between the two groups' general data (*P* > 0.05) (Table 1).

### 3.2. Comparison of T-Cell Subsets between the Two Groups

The levels of T-cell subsets (CD4 and CD8) did not differ statistically between the two groups (*P* > 0.05); however, the levels of CD4/CD8 in the observation group were significantly higher than those in the control group (*P* < 0.05) (Table 2).

### 3.3. Comparison of Serum IL-4, IL-8, IFN-*γ*, IL-17, and IgE Levels between the Two Groups

Children in the observation group had substantially higher serum IL-4 levels than those in the control group (*P* < 0.05); the observation group also had significantly higher serum IL-8 levels than those in the control group (*P* < 0.05); serum IFN-*γ* levels in the observation group were substantially lower than in the control group (*P* < 0.05); serum IL-17 levels in the observation group were substantially higher than in the control group (*P* < 0.05); children in the observation group had significantly higher serum IgE levels than children in the control group (*P* < 0.05) (Table 3).

## 4. Discussion

Bronchiolitis is a common lower respiratory tract infection in children, and it is characterized by involvement of bronchioles, with higher occurrence in children under 2 years of age. The clinical manifestations are wheezing, coughing, suffocation, and other symptoms. It is considered to be a risk factor for bronchial asthma and recurrent wheezing in children. The study found that the incidence of recurrent wheezing in children with bronchiolitis after treatment was as high as 85%, and the incidence of progression to asthma within 3 to 5 years was 35.83%. The respiratory syncytial virus is the most common infectious agent responsible for capillary bronchitis in children [10]. In addition to pathogen invasion into the bronchi of afflicted children, the disease's progression is linked to local spasms induced by the production of inflammatory factors in the affected organism [11]. According to clinically relevant research, multiple inflammatory cells of the body and inflammatory factors are involved in the development of capillary bronchitis [12].

Infants and children with respiratory syncytial virus capillary bronchitis had a 44 percent chance of developing asthma within the next 10 years, according to a study by Ma Hongtang et al. There is now widespread acceptance in academics that the pathogenesis of respiratory syncytial virus capillary bronchitis and asthma are analogous [13]. Moreover, researcher Qingqing Li et al. [14] showed that asthmatic patients have immunological dysfunction linked with alterations in T-cell subsets; therefore, in this study, we analyzed peripheral blood T-cell subsets CD4 and CD8 in children with respiratory syncytial virus capillary bronchitis.

According to the findings, children with respiratory syncytial virus capillary bronchitis have an immune impairment,. Although there was no statistically significant difference in CD4 and CD8 levels between the observation and control groups, the observation group's CD4/CD8 ratio was significantly higher. And this revealed that children with respiratory syncytial virus capillary bronchitis had a relative impairment in T suppressor cell activity and a relative hyperfunction of T helper cells, which was an essential mechanism leading to a change in key cytokines in the children patient [15]. According to a study by Wang Lan et al. [16], the pathogenesis of respiratory syncytial virus capillary bronchiectasis is a highly complex immunopathological process, and the severity of the disease is closely related to the immune response of the children.

Researchers Wenwen Ma et al. [17] discovered a correlation between IL-17 released by Thl7 and wheezing disease in infants and children. Its expression levels are significantly elevated in asthmatic patients' serum and lung tissues. Serum helper T cells 17 play an important role in some bacterial, viral, fungal, and parasitic infectious diseases, and the cytokines secreted are closely related to the occurrence of respiratory syncytial virus bronchiolitis. IFN-*γ* is a representative cytokine of serum helper T-17, and when the excretion of serum helper T-17 in children with respiratory syncytial virus bronchiolitis is affected, the expression level of IFN-*γ* in children is decreased. IL-17 is a cytokine secreted by serum helper T cells. In viral infection, IL-17 is considered to be a pathogenic factor because IL-17 is genetically homologous to herpes virus and can recruit concentrated granulocytes and cause an inflammatory response. In this study, we compared the serum IL-17 levels of the two groups. The results demonstrated that the serum IL-17 levels in the observation group were significantly higher than those in the control group, indicating that IL-17 is directly involved in the development of respiratory syncytial virus capillary bronchitis and that its level reflects the severity of this condition. Moreover, this indicates that children with respiratory syncytial virus capillary bronchitis have a relatively hyperfunctional Th17, which results in increased serum IL-17 production [18]. The potential explanation is that immune dysfunction is an important mechanism of childhood bronchiolitis, and helper T cells (Th cells) play an important immunoregulatory role in respiratory inflammatory diseases. IL-17 is secreted by CD4+ T cells and is an effector cell of Th17 cells, which can promote the activation of T cells and stimulate epithelial cells, endothelial cells, granulocyte-macrophage stimulating factor, etc. to mediate inflammatory responses. McGill et al. argued that the expression of IL-17 is increased in RSV-infected children, and that increased expression levels have a negative impact on the development of RSV-associated disease.

IFN-*γ* represents Th1 cytokines, while IgE can be used as a marker of Th2 cell immune response. In this study, the serum IFN-*γ* and IgE levels of the two groups were compared, and the results showed that the serum IFN-*γ* levels in the observation group were significantly lower than those in the control group; the serum IgE levels in the observation group were significantly higher than those in the control group, indicating that the Th1 function was suppressed in children with respiratory syncytial virus capillary bronchitis, with this being the primary cause of the reduced secretion of serum IFN-*γ* [19]; in children with capillary respiratory syncytial virus bronchitis, the Th1 function is inhibited, causing the Th2 function to be relatively hyperactive. In addition, eosinophils are important cells involved in type I allergy. When the body comes into contact with allergens for the first time, IgE is produced, and it can combine with eosinophils, resulting in a sensitizing characteristic. When the body is in contact with the same allergen again, these eosinophils that have developed sensitization characteristics can be gradually chemotactic into inflammatory areas by vascular endothelial cells under the promotion of chemokines and produce a large number of inflammatory mediators, accompanied by inflammatory cell infiltration, airway epithelial damage, increased mucus secretion, and other symptoms. Consequently, it results in a high response state in the airway and further leads to bronchitis. This is also attributable to the results of this study [20].

The hyperfunction of Th2 in children will boost the secretion of serum IL-4, and the increased secretion of IL-4 will promote the synthesis of IgE by the B lymphocytes of children. The increase in the level of IgE will aggravate the wheezing symptoms in children's airways [21]. According to a number of clinical research, serum IL-4 and IL-8, two typical factors released by Th2 cells, are considerably higher in asthmatic patients. We also compared serum IL-4 and IL-8 levels in two groups of children in this study; the results showed that serum IL-4 levels in the observation group were significantly higher than those in the control group, and serum IL-8 levels in the observation group were significantly higher than those in the control group. The current study's findings are consistent with previous studies, confirming the identical etiology of respiratory syncytial virus capillary bronchitis and asthma [22, 23]. They also support that Th1 function is suppressed, and Th2 cells are relatively more active in children with respiratory syncytial virus capillary bronchitis.

There are many studies on children with bronchiolitis, yet there is a paucity of reports on respiratory syncytial virus capillary bronchitis. It is currently known that the virus plays an important role in the onset of bronchiolitis and is also immensely detrimental to the health and growth of children. This study explored the changes of immune system factors in these children and provided certain ideas for the use and diagnosis of drugs by clinicians in the future. This study also had limitations, such as the analysis of just the children's serum samples at the time of admission and the omission of the children's indicators following treatment, which prevented a comprehensive evaluation of the dynamic changes in the children's peripheral blood T-lymphocyte subsets and serum indicators. More cases and comparative studies with centralized analysis are clinically required to more clearly illustrate the changes in T-cell subsets and serum IFN-*γ*, IL-17, and IgE levels in children with respiratory syncytial virus capillary bronchitis and their clinical significance.

In conclusion, the Th1/Th2 immune response imbalance caused by elevated CD4/CD8 levels in children with respiratory syncytial virus capillary bronchitis is comparable to the alterations identified in bronchial asthma, indicating a link between the pathophysiology of the two diseases. Children with respiratory syncytial virus capillary bronchitis have increased serum levels of IL-4, IL-8, IL-17, and IgE and decreased serum levels of IFN-*γ*, indicating that the levels of the aforementioned serum indicators may, to some extent, reflect the severity of the children's condition.

## Figures and Tables

**Table 1:** Comparison of general information in two groups [$\bar{\text{x}}\pm \text{s}$, *n*(%)].

	Observation group (*n* = 50)	Control group (*n* = 50)	*t*/*x*^2^	*P*
Gender			0.16	0.689
Male	27	25		
Female	23	25		
Age(month)	3-34	4-35		
Average age(month)	14.52 ± 5.27	14.62 ± 5.18	-0.096	0.924

**Table 2:** Comparison of T-cell subsets between the two groups ($\bar{\text{x}}\pm \text{s}$).

Group (case number)	CD4 (%)	CD8 (%)	CD4/CD8
Observation group (*n* = 50)	39.62 ± 6.41	21.83 ± 2.96	1.83 ± 0.33
Control group (*n* = 50)	38.14 ± 5.97	22.82 ± 3.80	1.63 ± 0.21
*t*	1.195	-1.453	3.616
*P*	0.235	0.149	<0.001

**(a):** 

Group (case number)	IL-4 (pg/ml)	IL-8 (pg/ml)
Observation group (*n* = 50)	49.83 ± 10.77	73.48 ± 8.51
Control group (*n* = 50)	32.35 ± 9.78	58.42 ± 10.04
*t*	8.496	8.091
*P*	<0.001	<0.001

**(b):** 

Group (case number)	IFN-*γ* (ng/l)	IL-17 (ng/l)	IgE (IU/ml)
Observation group (*n* = 50)	7.04 ± 1.85	26.03 ± 6.91	171.74 ± 58.16
Control group (*n* = 50)	8.96 ± 1.65	13.54 ± 5.16	43.93 ± 12.83
*t*	-5.477	10.241	15.174
*P*	<0.001	<0.001	<0.001

## Data Availability

All data generated or analysed during this study are included in this published article.
